The article "Topical Application of Premna integrifolia Linn on Skin Wound Injury in Rats Accelerates the Wound Healing Process: Evidence from In Vitro and In Vivo Experimental Models" was published in 2022. Journal: Evid Based Complement Alternat Med.

# Topical Application of *Premna integrifolia* Linn on Skin Wound Injury in Rats Accelerates the Wound Healing Process: Evidence from *In Vitro* and *In Vivo* Experimental Models

**DOI:** 10.1155/2022/6449550

**Published:** 2022-04-13

**Authors:** Saeed Ali Alsareii, Nasser A. N. Alzerwi, Mansour Yousef AlAsmari, Abdulrahman Manaa Alamri, Mater H. Mahnashi, Ibrahim Ahmed Shaikh

**Affiliations:** ^1^Department of Surgery, College of Medicine, Najran University, Najran, Saudi Arabia; ^2^Department of Surgery, College of Medicine, Majmaah University, Ministry of Education, Al-Majmaah City, Saudi Arabia; ^3^Department of Pharmaceutical Chemistry, College of Pharmacy, Najran University, Najran, Saudi Arabia; ^4^Department of Pharmacology, College of Pharmacy, Najran University, Najran, Saudi Arabia

## Abstract

**Background:**

When the skin and tissues within the body are injured, the healing process begins. Medicinal herbs have been used to cure wounds since time immemorial. The antimicrobial and antioxidant activity possessed by *P. integrifolia* may accelerate wound healing.

**Objectives:**

To assess the wound healing activity of Premna integrifolia extract (PIE) by employing in-vivo experimental animal models and an in-vitro migration scratch assay. Furthermore, to assess its cytotoxicity using the MTT assay.

**Methods:**

Wistar albino rats were used for the *in vivo* wound healing models. The animals were divided into four groups at random: Group I was untreated. Group II was vehicle control (ointment base). Group III was PIE ointment (5% W/W). Group IV was standard (povidone-iodine ointment) (5% W/W). The ointments were applied directly to the wounds as described above until they healed completely. The wound contraction percentage and tensile strength were calculated. The MTT test was used to determine the viability of the test extract against the fibroblast cells. The scratch assay was used *in vitro* to determine the wound healing potential of the test drug. *P* ≤ 0.05 values were considered statistically significant.

**Results:**

*Premna integrifolia* extract did not possess any noticeable cytotoxicity to the cell line and showed an IC_50_ of 185.98 *μ*g/ml. The wound contraction potential of PIE ointment-treated animals was considerably greater (*P* ≤ 0.001) on days 4, 8, 12, 16, and 20 when compared to the control group. The percentage of wound contraction on day 20 was 99.92% in PIE-treated animals compared to 83.23% in untreated animals. Compared to the untreated group, the duration of full epithelization was significantly (*P* ≤ 0.01) shorter in the test group. When compared to the incision control group, the animals treated with PIE ointment had significantly higher (*P* ≤ 0.001) tensile strength. In addition, animals given the test drug had a significant (*P* ≤ 0.001) increase in total protein and hydroxyproline. In the *in vitro* scratch assay, test drug-treated cells demonstrated greater cell migration. Histology images confirmed that the test drug-treated group had epithelial tissue proliferation and keratinization.

The article "Topical Application of Premna integrifolia Linn on Skin Wound Injury in Rats Accelerates the Wound Healing Process: Evidence from In Vitro and In Vivo Experimental Models" was published in 2022. Journal: Evid Based Complement Alternat Med.

**Conclusion:**

The current study found that *Premna integrifolia* improved wound healing activity both *in vitro* and *in vivo*. These findings indicate that *Premna integrifolia* extract has wound-healing potential and could be a viable source of nutraceuticals with wound-healing properties.

## 1. Introduction

A wound is a rupture in the continuity of a living tissue's cellular, functional, and anatomical properties caused by chemical, physical, thermal, immunological, or microbial assaults [1]. To restore the structural integrity of the damaged tissue, a sequence of activities must occur, including cell migration, proliferation, interaction, differentiation, bimolecular interactions, matrix component creation, and a complicated signaling network [2].

The regulation of the acute wound healing process is determined by interacting processes at the cellular, molecular, and extracellular matrix levels and concludes with wound closure in extended periods of time [3]. Physiological healing can be divided into three stages: inflammation, proliferation, and remodeling [4]. However, an asymmetry between metalloproteinases (MMPs) and the associated tissue inhibitors of metalloproteinase (TIMPs) may impede the healing process throughout the inflammatory phase, particularly during the tissue formation phase. Chronic wounds are used to characterize this type of injury [4, 5]. Although the mechanism underlying this chronic wound is complex, it is frequently linked to other comorbid disorders, such as diabetes, obesity, vascular insufficiency, or high blood pressure. Local hypoxia, bacterial colonization, and repeated ischemia-reperfusion damage, as well as cellular and systemic alterations, are the most common symptoms associated with chronic wounds [6].

Skin injury has been considered to be a complicated process. The current wound management strategies for resolving minor to severe injuries include irrigation, debridement, proteolytic enzymes, antibiotics, and tissue grafts, however, they have been linked to severe downsides, such as invasiveness and cost [7]. The emergence of antibacterial resistance combined with the high cost and slow rate of new antibiotic development increases wound-related mortality and morbidity. The rise of resistant bacterium strains, particularly those that cause wounds, such as *Pseudomonas* and *Acinetobacter* species that are multidrug-resistant, vancomycin-resistant *Staphylococcus aureus* (VRSA), and methicillin-resistant *Staphylococcus aureus* (MRSA), remains a global public health concern. As a result, wound infection continues to be the most common cause of nonhealing wounds and continues to be a considerable burden for both patients and caregivers [8, 9]. Apart from being expensive, the drugs utilized in the management of wounds pose issues, such as hypersensitivity reactions and resistance [10]. Herbal medicines can solve the adverse effects, costs, and antimicrobial resistance issues. The antimicrobial activity possessed by the phytoconstituents in herbal extracts may aid in wound healing [11]. The effectiveness of antimicrobials in wound healing is well-established and reinforces their role in accelerating wound healing with either systemic or topical use [10–12].

The article "Topical Application of Premna integrifolia Linn on Skin Wound Injury in Rats Accelerates the Wound Healing Process: Evidence from In Vitro and In Vivo Experimental Models" was published in 2022. Journal: Evid Based Complement Alternat Med.

Since the dawn of time, medicinal herbs have been utilized to treat wounds. Natural products, particularly plant secondary metabolites, such as isoprenoids, phenolics, and alkaloids, have been shown to be the most effective sources of novel wound healing agents [13]. *Premna integrifolia* Linn. (Lamiaceae) is a common shrub with 40 species found in tropical and subtropical locations around the world, including the United States, India, Australia, Bangladesh, and China. Although this genus has several species, only two of them, *P. latifolia* and *P. integrifolia,* are known to have medicinal properties [14].

Several diseases, including bronchitis, diabetes, edema, chyluria, dyspepsia, inflammation, liver problem, constipation, piles, and fever can be treated with the roots of *P. integrifolia* [15]. Anticoagulant, antiarthritic, antihyperglycemic, and antimicrobial characteristics have also been reported for the plant [15]. It protects against cardiovascular diseases since it contains alkaloids and iridoid glycosides [16].

*P. integrifolia* ethanolic extract exhibits potent antidiabetic, analgesic, antibacterial, antiulcer, and antioxidant properties [15]. *P. integrifolia* leaf extracts were found to have hepatoprotective properties against carbon tetrachloride and paracetamol-induced liver damage [15]. However, no research has been done on the plant's effectiveness in wound healing. The current study was carried out to evaluate the wound-healing property of *P. integrifolia,* utilizing the incision wound model and excision wound model, in perspective of its anti-inflammatory and antibacterial characteristics.

## 2. Materials and Methods

### 2.1. *Premna integrifolia* Extract

The standardized extract of *Premna integrifolia* was procured from Vital Herbs Z-26/27 Commercial Enclave, Uttam Nagar, New Delhi, India.

The article "Topical Application of Premna integrifolia Linn on Skin Wound Injury in Rats Accelerates the Wound Healing Process: Evidence from In Vitro and In Vivo Experimental Models" was published in 2022. Journal: Evid Based Complement Alternat Med.

### 2.2. Ointment Formulation

A simple ointment (British Pharmacopoeia) was prepared using white soft paraffin, cetostearyl alcohol, hard paraffin, and wool fat [17].

Procedure: hard paraffin (5 g) was melted in a beaker over a water bath to make the 100 g simple ointment base. The remaining ingredients were added in the descending order of melting point: cetostearyl alcohol (5 g), white soft paraffin (85 g), and wool fat (5 g). All of the ingredients were melted in a water bath while being constantly stirred until they were completely homogeneous. The mixture was taken off the heat and stirred until it was completely cool. Five grams of *P. integrifolia* extract were mixed with a portion of the simple ointment base to make a 5% (w/w) ointment. The rest of the simple ointment base was gradually added and thoroughly mixed in. The prepared ointment was stored in a clean and dry container, away from heat. The ointment was used for topical application on the wounds for 20 consecutive days during the experiment.

### 2.3. Animals

Male and female Wistar albino rats (≈200 g) were maintained under typical ambient conditions of humidity and temperature (25 ± 0.5 C) and a 12 h light/dark cycle. The rats were given a conventional pellet diet and free access to water. The animal research was carried out at the institute with the Najran University Scientific Research Ethical Committee's approval, vide number 443-41-49631-DS.

### 2.4. Acute Dermal Toxicity

The goal of the study was to figure out what the therapeutic dose of the standardized extract should be. The extract's acute cutaneous toxicity was tested by applying an ointment containing extract at the highest concentrations of 5% (w/w) to the rats' shaved backs. The study was conducted in accordance with OECD Guidelines No. 434 [18].

### 2.5. Wound Healing Activity

With six animals in each group, the animals were divided into four major groups: control, base, test, and standard. The control group was not given any treatment. The base (vehicle) control group received only the ointment base. The test group was given ointment with a high concentration of extract (5% w/w) mixed into a simple ointment base. Cipladine (5% w/w povidone-iodine ointment) was used on the control group.

### 2.6. Excision Wound Model

The animals were divided into four groups at random: Group I: untreated excision; Group II: vehicle control (ointment base); Group III: PIE ointment (5% W/W); Group IV: standard (povidone-iodine ointment 5% W/W). Ketamine (0.5 ml/kg b. w. i.p.) was used to anesthetize the rats. On the shaved backs of the rats, a full-thickness excision wound of circular area (about 250 mm^2^) and 2 mm depth was made 30 minutes after the injection of ketamine. Day 0 was designated as the day of the wounding (Figure 1). The topical application of the ointments as indicated above was used to treat the wounds until they were totally healed. On days 0, 4, 8, 12, 16, and 20, the wounds were observed, and the area of the wound and the mean percent wound contraction were assessed. The number of days required for the dead tissue to fall without any remaining raw wound was used to calculate the epithelization duration [19].

The article "Topical Application of Premna integrifolia Linn on Skin Wound Injury in Rats Accelerates the Wound Healing Process: Evidence from In Vitro and In Vivo Experimental Models" was published in 2022. Journal: Evid Based Complement Alternat Med.

### 2.7. Wound Healing Rate [20]

Wound healing rate is given by

(1) $$\begin{array}{c} \%\text{ of wound closure}=\frac{\text{wound area on day }0-\text{wound area on day }n}{\text{wound area on day }0}\times 100. \end{array}$$

## 3. Estimation of Biochemical Markers

### 3.1. Hydroxyproline Estimation

The hydroxyproline content of resected wound tissues was determined on day 20 of the experiment. The tissue samples were dried in a hot air oven at 60°C, and thereafter, they were hydrolyzed for four hours at 130°C in 6 N HCl. The hydrolysates were neutralized to pH 7.0 and oxidized with Chloramine-T for 20 minutes. The reaction was stopped after 5 minutes by adding 0.4 M perchloric acid and developing color with Ehrlich's reagent at 60 C. The materials were examined in an ultraviolet spectrophotometer at 557 nm after complete stirring. The hydroxyproline concentration of the tissue samples was determined using a pure L-hydroxyproline standard curve [21].

### 3.2. Protein Estimation

Protein estimation was determined on day 20 of the experiment. Tissue specimens were homogenized overnight in 0.1 N NaOH. The homogenate (2 mL) was placed in a vial and centrifuged for 15 minutes at 5000 rpm. 1 mL of supernatant was added to 1 mL of reagent (50 mL of 2% Na_2_CO_3_ in 0.1 N NaOH + 2 mL of 0.5 percent CuSO_4_ in 1% sodium potassium tartrate) in a separate vial. At room temperature, the samples were incubated for 15 minutes. Each sample received 100 mL of Folin–Ciocalteau reagent, which was left at room temperature for 30 minutes. A UV–vis spectrophotometer was used to measure absorbance at 670 nm within 30 minutes [22].

### 3.3. Incision Wound Model

Ketamine (0.5 ml/kg b. w. i.p.) was used to anesthetize the rats. Thirty minutes after the rats were given ketamine, sterilized scalpels were used to make 6 cm long and 2 mm deep incision wounds on their shaved backs (figure 1(b)). The skin was held together by stitching it at 0.5 cm intervals with black silk. Stitching was done with surgical thread (number. 000) and a curved needle (no. 9). The continuous thread on both wound edges was tightened to ensure that the wounds were properly closed. The wounds of the animals in each group were treated for 10 days with the topical treatment of the ointments as indicated above. The day of the wounding was counted as day 0. On the eighth postwounding day, the sutures were removed, and the tensile strength of the skin, defined as the weight in grams necessary to tear open the skin/wound, was determined using a tensiometer on day 10 [23].

The article "Topical Application of Premna integrifolia Linn on Skin Wound Injury in Rats Accelerates the Wound Healing Process: Evidence from In Vitro and In Vivo Experimental Models" was published in 2022. Journal: Evid Based Complement Alternat Med.

### 3.4. MTT Assay

The MTT test was used to determine whether the test extract was viable against L929 Mouse transformed fibroblast cell line. Different concentrations of the test extract (50–250 *μ*g/ml) were added to the fibroblast cell lines. The fibroblast cell lines were cultured for 24 hours in DMEM. After that, 10 *μ*l MTT (3-(4, 5-dimethyl-thiazol-2-yl)-2, 5-diphenyl tetrazolium bromide) was added to each well and allowed to sit for 2 hours. After dissolving the formazan crystals with dimethyl sulfoxide (DMSO), absorbance was measured at 570 nm in a microtitre plate [24]. Cisplatin is the known standard cytotoxic drug, and it was used as a control to compare the results of the test drug.

### 3.5. *In Vitro* Wound Healing Activity

The trypsinized cells were aspirated into a 5 ml centrifuge tube. Centrifugation at 300 x g yielded a cell pellet. The cell count was adjusted in each well of the 12-well plate using DMEM. Then, 1 ml DMEM containing 100 *μ*l of the cell suspension was added, and the plate was incubated at 37°C and 5% CO_2_ for 24 hours to achieve 100% confluence as a monolayer. A new 200 *μ*l pipette tip was used to scratch the monolayer gently and slowly over the center of the well. To remove the detached cells, gently wash the well twice with medium after scratching. Refill the well with fresh media after washing the cells twice with 1x Phosphate Buffered Saline (PBS). The PBS was sucked out. With 1 ml of new medium, 25 *μ*l of varied test concentrations from the stock of test medications were introduced to the appropriate wells. The images of the scratched monolayers were obtained at different time intervals of 0 hours, 12 hours, and 24 hours, followed by a 24-hour incubation of the plate at 37°C and 5% CO_2_. By measuring the gap distance at 4X resolution using MagVision Software, the gap distance was quantified [25].

The rate of migration was calculated using the below formula:

(2) $$\begin{array}{c} Rm=\frac{\left(W_{i}-W_{t}\right)}{T}, \end{array}$$

where *Rm*: rate of cell migration (*μ*m/h); *W*_*i*_: initial wound width (*μ*m); *W*_*t*_: final wound width (*μ*m); *T*: duration of migration (hours)

## 4. Antibacterial and Antifungal Activity

### 4.1. Agar-Well Diffusion Method

Petri plates containing 25 ml of optimized media were seeded using a glass rod with 24 hr-old cultures of *Candida albicans* strains for assessing antifungal activity and *Escherichia coli* (Gram +ve) and *Bacillus cereus* (Gram −ve) strains for assessing antibacterial activity. The spread plate method was followed, and the wells were made using a well-borer. A stock concentration of 100 mg in 1 ml and a standard drug (Itracanozole and ciprofloxacin) of 30 µl were used. The plates were then incubated at 37°C for 24 hours. The antimicrobial activity was confirmed by measuring the diameter of the inhibition zone formed around the well.

The article "Topical Application of Premna integrifolia Linn on Skin Wound Injury in Rats Accelerates the Wound Healing Process: Evidence from In Vitro and In Vivo Experimental Models" was published in 2022. Journal: Evid Based Complement Alternat Med.

### 4.2. Histological Examination

At the conclusion of the experiment, skin biopsies were taken from the rats and preserved in a buffered formaldehyde solution (10% v/v). Tissue samples were treated and fixed in paraffin wax on a regular basis. Hematoxylin and eosin were used to stain the longitudinal sections (5 mm) of healed lesions. On coded slides, the microscopic examination was done blindly using a light microscope.

### 4.3. Statistical Analysis

The data was statistically analyzed using GraphPad Prism® version 5.01 (GraphPad Software, USA) using one-way analysis of variance, followed by Tukey's post hoc test. *P* 0.05 was used as a cut-off point for statistical significance.

## 5. Results

### 5.1. Acute Dermal Toxicity Test

There were no signs of inflammation or edema after applying a 5% w/w ointment dose during the first 24 hours. In addition, 14 days after topical application of the PIE ointment, no mortality or signs of toxicity were observed.

### 5.2. MTT Assay

Phytochemicals have long been researched for their therapeutic characteristics, however, their cytotoxic effects on the cell type of interest are often overlooked. However, there has been an increasing trend to examine this crucial component in recent years. The MTT assay was used to check the cytotoxicity of the test extract against a fibroblast cell line. The test extract was less cytotoxic to the normal cell line than the control drug cisplatin. The cell line treatment with various doses of test extract had no discernible cytotoxicity and showed an IC_50_ of 185.98 *μ*g/ml. However, at a concentration of 250 *μ*g/ml of test extract, a little reduction in cell viability was observed (Figure 2). These results showed that *P. integrifolia* extract was not cytotoxic and that its medicinal potential may be investigated further. In contrast, cells treated with cisplatin showed maximum toxicity. Cisplatin inhibits cell proliferation by a cytotoxic mechanism, characterized by DNA damage and the modulation of oxidative stress. Exposure to oxidative stress can upset regular biological functions. Cisplatin also induces reactive oxygen species that trigger DNA damage, leading to cell death. Cell death occurs upon the immediate activation of numerous signaling pathways.

The article "Topical Application of Premna integrifolia Linn on Skin Wound Injury in Rats Accelerates the Wound Healing Process: Evidence from In Vitro and In Vivo Experimental Models" was published in 2022. Journal: Evid Based Complement Alternat Med.

### 5.3. Effect of the Standardized Extract of *Premna integrifolia* on Percentage Wound Contraction and Epithelialization Period

Table 1 and Figure 3 show the results of wound-healing activity using the excision wound model. The percentage wound-healing values shown in the table are for excision control, base, test extract, and the standard group at 0, 4, 8, 12, 16, and 20 days. The wound-contracting ability of animals treated with the ointment containing 5% (w/w) test extract was shown to be considerably higher (P 0.001) on days 4, 8, 12, 16, and 20 when compared to the excision control group (Figure 4). On day four after wounding, the control group animals had firm thrombus edema and exudates on the wound area (group I), while a comparatively soft thrombus with a decrease in inflammation and no noticeable discharge was observed in the PIE ointment (group III) and standard treated group (group IV). The generation of reddish connective tissue was detected in the animals of groups III and IV on day eight. In group IV, however, it was noticed earlier (on the eighth day after wounding) than in group III. In comparison to group I, the animals treated with standard and PIE ointment significantly (P 0.001) improved wound-healing effects in the rat models and aided in wound contraction from day 4 to day 20.

The complete epithelization period for group I animals was 17 days, while epithelization times for group III and group IV animals were 11 and 8.6 days, respectively. In comparison to the untreated group, the full epithelization duration was significantly (P 0.01) shorter in groups III and IV. The wound-healing effect of PIE ointment was found to be comparable to that of the commercially available 5% w/w povidone-iodine ointment (standard).

### 5.4. Hydroxyproline Content

The animals treated with the test extract exhibited significantly (71.72 ± 0.79 *μ*g/100 mg of tissue) higher hydroxyproline content than the excision control. The standard control group showed 90.41 ± 0.9241 *μ*g/100 mg of tissue [figure 5(a)].

### 5.5. Protein Estimation

The levels of total protein in the tissue were found to be 131 ± 3.26, 107.2 ± 2.45, 78.17 ± 2.3, 67.50 ± 2.26 *μ*g/100 mg of issue in the standard, test extract, base, and excision control groups, respectively. The animals treated with the test and standard drug have shown a significant (*P* < 0.001) increase in total protein level compared with the excision control animals [figure 5(b)].

The article "Topical Application of Premna integrifolia Linn on Skin Wound Injury in Rats Accelerates the Wound Healing Process: Evidence from In Vitro and In Vivo Experimental Models" was published in 2022. Journal: Evid Based Complement Alternat Med.

### 5.6. Incision Wound Study

The tensile strength of the incision wound was used to assess the influence of the wound-healing activities in this model. The results are provided as the mean weight in Gram ± SEM, necessary to burst open the sutured incision (Table 2 and Figures 6 and 7). When compared to the incision control group, the animals treated with PIE ointment had considerably higher (*P* = 0.001) tensile strength. (P 0.001) tensile strength.

### 5.7. *In Vitro* Wound-Healing Cell Migration Assay

Scratch assay is a frequently used *in vitro* technique for determining a compound's wound-healing potential. In the current study, the mouse fibroblast cell line was treated with *Premna integrifolia* for 24 hours. Cell migration was captured at different time intervals of 0 hrs, 6 hrs, 12 hrs, and 24 hrs. The results showed that the PI extract (18 *μ*g/mL) filled the scratch gap by 87.89 percent in 24 hours.  Table 3 shows the percentage of wound closure at various time periods in untreated, extract-treated, and standard drug-treated cells. When compared to the control, the test extract caused the fibroblast cells to migrate, resulting in a higher percentage of wound closure. At 24 hours, 96.53% of the gap in the cells treated with the standard drug had been closed, which was almost similar compared to the test drug. In the standard and the extract-treated cells, the images demonstrate greater cell migration (Figure 8).

### 5.8. *In Vitro* Antimicrobial Activity

The data obtained from the standard antimicrobial assay of *Premna integrifolia* were compared with that of the standard drugs. The antimicrobial assay test results showed a promising outcome when compared to that of standard antimicrobial agents. The results showed that *E. coli* (Gram −ve), *B. cereus* (Gram +ve), and *C. albicans* strains were susceptible to the tested drug with the inhibition zone diameter of 20 mm, 07 mm, and 9 mm, respectively (Table 4 and Figure 9).

### 5.9. Histopathological Study

On the twentieth day, the histological investigations of the skin in the excision wounds were done, and the histopathological features of the tissue from all groups of animals are depicted in Figure 10. Animals in group I (A) (excision control) had inflammatory cells, decreased collagen fibers, fibroblast cells, and blood vessels, as well as apparent scar tissue. Group II (B) (base treatment) exhibited necrotic cells and fewer collagen fibers and blood vessels. However, as compared to the control, group III (C) (PIE ointment) revealed significantly more fibroblast cells, blood vessels, and well-organized collagen fibers. Group IV (D) (standard) demonstrated complete tissue regeneration as evidenced by increased fibroblast cells, collagen fibers, and blood vessels, as well as decreased inflammatory cells. Both the extract ointment-treated and standard groups demonstrated epithelial tissue proliferation and keratinization.

The article "Topical Application of Premna integrifolia Linn on Skin Wound Injury in Rats Accelerates the Wound Healing Process: Evidence from In Vitro and In Vivo Experimental Models" was published in 2022. Journal: Evid Based Complement Alternat Med.

## 6. Discussion

Wound-healing is a sophisticated process that takes place when the skin and other soft tissues of the body are damaged. Wound-healing is a dynamic process that involves numerous chemical pathways with the goal of returning the wounded cellular structure to its original form [26]. The conventional wound-healing cascade consists of three sequential and overlapping steps: inflammation, proliferation, and remodeling [27].

To further understand the extended usage of crude plant extracts or purified secondary metabolites in wound healing, a variety of *in vitro* investigations have been conducted. Several medicinal plants have been identified as medicinally relevant and important in both traditional and modern scientific studies [28]. *P. integrifolia* is an edible plant and has culinary uses. Its leaves are eaten by the inhabitants of the Coromandel coast, India. In Vietnam, the aromatic leaves are used to cook in some braise or stir fry dishes [29]. Thus, the consumption of this plant may also help heal gastric ulcers. Although *P. integrifolia*'s medical benefits have been known for decades, they are yet to be scientifically verified.

In the current study, we used *in vitro* assays and *in vivo* animal models to examine the wound-healing characteristics of *Premna integrifolia*.

In the current investigation, the topical administration of PIE (5% w/w) ointment promoted wound healing in both excision and incision wound types in rats. Recent research has suggested that triterpenoids, flavonoids, and tannins play an important role in wound healing through various mechanisms, including wound contraction, increased rate of epithelialization, and prevention of secondary bacterial infection [30, 31]. Previous studies on *Premna integrifolia* found the presence of sterols, flavonoids, tannins, and saponins, all of which aid in wound healing.

In our investigation, the test extract-treated groups exhibited a larger area of wound contraction than the excision control and ointment base groups. Furthermore, the tensile strength of PIE ointment was higher than the incision control animals. It could be related to increased fibroblast activity, increased collagen synthesis, antioxidant, anti-inflammatory [32], and antibacterial properties of the plant. In the current study, the antimicrobial activity of PIE was assessed, and it showed good antibacterial and antifungal potential.

Wound contraction shortens healing time by lowering wound size and the volume of extracellular matrix needed to repair the injury. The wound-healing property of the PIE was parallel to that of povidone-iodine ointment, which is used as a standard treatment for wound-healing. Povidone-iodine is a well-known antibacterial medication that is used to prevent persistent wound infections.

The article "Topical Application of Premna integrifolia Linn on Skin Wound Injury in Rats Accelerates the Wound Healing Process: Evidence from In Vitro and In Vivo Experimental Models" was published in 2022. Journal: Evid Based Complement Alternat Med.

Collagen is an extracellular protein found in the granulation tissue of a regenerating wound, assisting wound resilience and tissue matrix integrity [33, 34]. Controlled synthesis and the deposition of new collagen and its maturation are essential for wound healing [35]. In the current study, wound contraction was substantially higher in PIE-treated animals compared to the control group, which could be attributable to increased collagen synthesis. It could be related to the presence of phenolic compounds [25, 28], however, flavonoids may also help prevent secondary wound infections because they have antiviral and antibacterial properties [36]. This study focuses on hydroxyproline levels as a biochemical measure of collagen turnover. Significantly higher (*P* ≤ 0.001) hydroxyproline content in the granulation tissue of PIE ointment-treated rats shows an elevated level of collagen content, which leads to rapid wound-healing, and this significant finding could be attributed to the presence of flavonoids [37]. Subsequently, the tensile strength of the treated wounds increased, which could be attributed to higher collagen levels and collagen fiber stabilization [38].

There was no indication of pus build-up, polymorphonuclear cell infiltration, fibrin deposition, or edema in animal lesions in the drug-treated group. Wound infection is the most common cause of delayed healing of skin wounds. Some of the most common bacteria that cause wound infection are *P. aeruginosa*, *E. coli*, *S. pyogenes*, *S. aureus*, and *Corynebacterium sp*. [39]. PIE previously demonstrated antibacterial action against *B. subtilis*, *S. lutea*, *E. coli*, *Pseudomonas sp., X. campestris*, and *K. pneumoniae* [40]. In the present study, PIE exhibited good antibacterial and antifungal activity, which might be one of the mechanisms responsible for its wound-healing potential. It has been previously reported that plants rich in polyphenols exhibit significant antibacterial activity [41, 42].

The *in vitro* MTT assay is well-known for testing the cytotoxicity of test drugs against fibroblast cell lines. In this experiment, fibroblast cells were treated with PIE at various concentrations (50–250 *μ*g/ml) and showed minimal or very minor toxicity to the fibroblast cells [43].

In the scratch-healing assay, scratching forms a “wound gap” in a cell monolayer, and the “healing” of this breach by cell proliferation and migration toward the center of the gap is recorded and frequently analyzed [44]. Factors affecting cell migration and/or proliferation can cause the gap to “heal” at a quicker or slower rate. This assay is easy to use and affordable, and the experimental settings can be simply changed to suit varied needs.

The article "Topical Application of Premna integrifolia Linn on Skin Wound Injury in Rats Accelerates the Wound Healing Process: Evidence from In Vitro and In Vivo Experimental Models" was published in 2022. Journal: Evid Based Complement Alternat Med.

In the present study, when fibroblast cells were treated with *P. integrifolia* extract, we found that they migrated better toward the artificially created wound. It indicates that the extract hastens wound healing by causing fibroblast migration. A similar study on *A. saccata* leaves extract found that its methanolic extract stimulated the migration of fibroblasts while also increasing the expression of wound-healing genes [28].

One of the primary benefits of the scratch method is that it approximates cell mobility *in vivo* to some extent. Endothelial cells (ECs) migrate into the wound region to mend the wound. Furthermore, migration patterns mimic the behavior of these cells during *in vivo* migration, whether as a loosely connected population (e.g., fibroblasts) or as sheets of cells (e.g., epithelium and ECs). Another advantage of this experiment is its ability to investigate extracellular matrix and cell-cell interactions as regulators of cell migration [44].

## 7. Conclusion

The present research demonstrated that *Premna integrifolia* enhanced wound-healing activity *in vitro* and *in vivo*. The obtained results showed that the application of PIE on wounds induced considerable wound contraction and accelerated healing. Furthermore, the extract was determined to have good antibacterial activity and had no cytotoxic effects. These findings show that *Premna integrifolia* extract possesses wound-healing potential and could be a viable source for isolating natural wound-healing phytochemicals. However, further clinical trials are warranted to extrapolate the results of this study in human beings.

### 7.1. Limitations, Economic Aspects, and Applied Suggestions

In the field of regenerative medicine for wound repair, most wounds are currently treated with supportive measures, such as appropriate wound dressing, maintaining hygiene, and prophylactic antibiotic use rather than drugs that innately boost the healing process. Drugs for wound healing should ideally be designed so that they are effective and provide quick results, reduce patient morbidity and suffering, and, most importantly, are cost-effective. *Premna integrifolia* ointment shows excellent promise for the future of wound healing while also being cost-effective. The animal models for wound healing are not devoid of their limitations. There are differences in the anatomy and physiology of rodents and human skin. The architecture of human skin is not reflected by the loose skin and dense hair on the rodent skin. There is no single animal model that can capture the heterogeneity and complexity of human wounds. The ultimate challenge remains to be the reproducibility and translation of preclinical data into clinical reality. Rat wounds heal primarily through contraction, reducing the importance of re-epithelialization and granulation unless a splinting technique is used, and they are less tractable genetically than mice.

The article "Topical Application of Premna integrifolia Linn on Skin Wound Injury in Rats Accelerates the Wound Healing Process: Evidence from In Vitro and In Vivo Experimental Models" was published in 2022. Journal: Evid Based Complement Alternat Med.

## Figures and Tables

**Figure 1:** (a) Circular excision wound on day 0. (b) Linear incision wound on day 0.

**Figure 2:** Pictographs. (a) Untreated. (b) *Premna integrifolia* extract (250 *μ*g/ml). (c) Cisplatin.

**Figure 3:** Photos depicting the effect of PIE ointment on excision wound model across different stages of the study.

**Figure 4:** The percentage contraction of the wound area was employed as an evaluation criterion for *in vivo* wound-healing activity using an incision wound model. Values are expressed as mean ± SEM for 6 animals per group. ^*∗*^*P* < 0.01. ^#^*P* < 0.001 compared with controls (ANOVA followed by post hoc tests for multiple comparisons).

**Figure 5:** (a) The hydroxyproline content of various animal groups' granulation tissues. (b) Protein content in the granulation tissues of different animal groups.

**Figure 6:** The effect of PIE ointment on tensile strength in incision wound model in Wister rats.

**Figure 7:** Photos depicting the effect of PIE ointment on the incision wound model across different stages of the study. (a) Wound suturing on day 0. (b) Wound-healing on day 8. (c) Wound-healing on day 12. (d) Wound-healing on day 16. (e) Tensile strength of test drug-treated animal wound on day 20 (wound did not open after applying 1090 g of weight). (f) Tensile strength of control animal wound on day 20 (sutured wound opened after applying 768 g of weight).

**Figure 8:** Microscopical photos illustrating *Premna integrifolia*'s ability to heal wounds *in vitro*. Images were taken at 0, 6, 12, and 24 hours after the mice fibroblast cells were cultured in the presence or absence of the test and standard drugs.

**Figure 9:** Antimicrobial activity of *P. integrifolia* against *C. albicans*: control itraconazole (a) and drug-treated (b). *B. cereus*: control ciprofloxacin (c) and drug-treated (d). *E. coli*: control ciprofloxacin (e) and drug-treated (f).

**Figure 10:** Histopathology analysis of newly healed tissue on day 20 post-treatment with PIE ointment. (a) Group I (excision control). (b) Group II (base treatment). (c) Group III (PIE ointment). (d) Group IV (Standard-Povidone-Iodine).

The article "Topical Application of Premna integrifolia Linn on Skin Wound Injury in Rats Accelerates the Wound Healing Process: Evidence from In Vitro and In Vivo Experimental Models" was published in 2022. Journal: Evid Based Complement Alternat Med.

**Table 1:** Effect of PIE on wound diameter, wound area, and percentage of wound contraction in an excision wound model.

Groups	Wound diameter (mm)						Area (mm sq)						Percentage wound contraction (%)					
	D0	D4	D8	D12	D16	D20	D0	D4	D8	D12	D16	D20	D0	D4	D8	D12	D16	D20

Excision (control)	24.5 ± 0.58	23.7 ± 0.5	22.5 ± 0.5	15.5 ± 0.58	12.5 ± 0.58	10 ± 0.82	471.4 ± 22.2	442.9 ± 18.4	397.6 ± 20.4	188.8 ± 14.5	122.9 ± 11.3	78.9 ± 8.83	0	5.8 ± 0.87	15.51 ± 2.89	59.88 ± 3.54	73.89 ± 2.71	83.23 ± 2.97
Base	24.7 ± 0.5	23.5 ± 0.58	22.2 ± 0.43	13 ± 0.82	12.5 ± 1.29	8 ± 0.82	481 ± 19.2	433.7 ± 21.3	388.8 ± 17.7	133.1 ± 16.67	123.6 ± 12.4	50.6 ± 6.63	0	9.64 ± 1.34	19.11 ± 2.12	72.30 ± 3.57	74.13 ± 5.28	89.46 ± 2.13
Extract (PIE)	25 ± 0.5	21.5 ± 0.58	17.5 ± 1.12	10.5 ± 1.29	4 ± 1.41	0.5 ± 0.58	481 ± 19.2	363.1 ± 19.5	241.4 ± 25.5	87.5 ± 11.3	13.7 ± 2.8	0.4 ± 0.11	0	24.43 ± 3.32^*∗*^	49.70 ± 6.32^*∗∗*^	81.75 ± 4.6^*∗∗*^	97.15 ± 1.58^*∗∗*^	99.92 ± 0.09^*∗∗*^
STD (povidone-iodine)	24.5 ± 0.58	20 ± 1.41	15 ± 0.71	8.75 ± 0.96	2.7 ± 0.96	0	471.4 ± 22.2	315.2 ± 20.4	177 ± 19.2	60.6 ± 9.47	6.5 ± 0.9	0.0	0	32.75 ± 5.85^*∗∗*^	62.28 ± 5.49^*∗∗*^	87.20 ± 2.31^*∗∗*^	98.64 ± 0.90^*∗∗*^	100 ± 0^*∗∗*^

Values are expressed as mean ± SEM for 6 animals per group. ^*∗*^*P* < 0.01. ^*∗∗*^*P* < 0.001 compared with controls (ANOVA followed by post hoc tests for multiple comparisons).

**Table 2:** Effect of PIE on tensile strength in the incision wound-healing model.

S. no.	Groups	Tensile strength (gm)

1	Incision control	768.0 ± 4.041
2	Base	862.5 ± 3.030
3	Extract (PIE)	1090 ± 16.09^*∗∗∗*^
4	STD (povidone-iodine)	1204 ± 12.39^*∗∗∗*^

**Table 3:** The percentage of cell migration (wound closure) of STD and test samples at different time intervals.

S. no	Test sample	Duration	Cell migration in *μ*m	Percentage wound closure (24 h)

1	Untreated	12 hours	5.08	16.90%
		24 hours	4.589	

2	Standard drug	12 hours	15.12	96.53%
		24 hours	21.65	

3	*Premna integrifolia*	12 hours	21.44	87.89%
		24 hours	22.07	

**Table 4:** Antimicrobial activity of test drug as depicted by the zones of inhibition (mm).

*Escherichia coli* (Gram −ve)				*Bacillus cereus* (Gram +ve)			*Candida albicans* (fungi)		

Control (ciprofloxacin): 29 mm				Control (ciprofloxacin): 22 mm			Control (Itraconazole): 13 mm		
Test drug	Conc. 1	Conc. 2	Conc. 3	Conc. 1	Conc. 2	Conc. 3	Conc. 1	Conc. 2	Conc. 3
*Premna integrifolia*	0 mm	0 mm	20 mm	0 mm	0 mm	7 mm	0 mm	7 mm	9 mm

## Data Availability

The data related to this research are included in the Results section.

## References

[1] Mulkalwar S., Behera L., Golande P., Manjare R., Patil H. (2015). Evaluation of wound healing activity of topical phenytoin in an excision wound model in rats. *International Journal of Basic & Clinical Pharmacology*.

The article "Topical Application of Premna integrifolia Linn on Skin Wound Injury in Rats Accelerates the Wound Healing Process: Evidence from In Vitro and In Vivo Experimental Models" was published in 2022. Journal: Evid Based Complement Alternat Med.

[2] Shrimanker M., Patel N., Modi H., Dave R. (2013). A review: screening models for wound healing activity in animals. *American Journal of PharmTech Research*.

[3] Stephens P., Caley M., Peake M. (2013). Alternatives for animal wound model systems. *Methods in Molecular Biology*.

[4] Iorio V., Troughton L. D., Hamill K. J. (2015). Laminins: roles and utility in wound repair. *Advances in Wound Care*.

[5] Tyavambiza C., Dube P., Goboza M., Meyer S., Madiehe A. M., Meyer M. (2021). Wound healing activities and potential of selected african medicinal plants and their synthesized biogenic nanoparticles. *Plants*.

[6] Schreml S., Szeimies R. M., Prantl L., Karrer S., Landthaler M., Babilas P. (2010). Oxygen in acute and chronic wound healing. *British Journal of Dermatology*.

[7] Dreifke M. B., Jayasuriya A. A., Jayasuriya A. C. (2015). Current wound healing procedures and potential care. *Materials Science and Engineering: C*.

[8] Sandar W.-P., Saw S., Kumar A. M. V., Camara B. S., Sein M.-M. (2021). Wounds, antimicrobial resistance and challenges of implementing a surveillance system in Myanmar: a mixed-methods study. *Tropical Medicine and Infectious Disease*.

[9] DeLeo F. R., Chambers H. F. (2009). Reemergence of antibiotic-resistant *Staphylococcus aureus* in the genomics era. *Journal of Clinical Investigation*.

[10] Lipsky B. A., Dryden M., Gottrup F., Nathwani D., Seaton R. A., Stryja J. (2016). Antimicrobial stewardship in wound care: a position paper from the British society for antimicrobial chemotherapy and European wound management association. *Journal of Antimicrobial Chemotherapy*.

[11] Ravishankar K., Kiranmayi G. V. N., Prasad Y. R., Devi L. (2018). Wound healing activity in rabbits and antimicrobial activity of Hibiscus hirtus ethanolic extract. *Brazilian Journal of Pharmaceutical Sciences*.

[12] Madaan R., Kumar S., Bansal G., Sharma A. (2011). Estimation of total phenols and flavonoids in extracts of Actaea spicata roots and antioxidant activity studies. *Indian Journal of Pharmaceutical Sciences*.

[13] Pérez M., Robres P., Moreno B. (2021). Comparison of antibacterial activity and wound healing in a superficial abrasion mouse model of *Staphylococcus aureus* skin infection using photodynamic therapy based on methylene blue or mupirocin or both. *Frontiers of Medicine*.

[14] Mali P. (2015). Premna integrifolia L.: a review of its biodiversity, traditional uses and phytochemistry. *Ancient Science of Life*.

[15] Mali P. (2016). Pharmacological potentials of Premna integrifolia L. *Ancient Science of Life*.

The article "Topical Application of Premna integrifolia Linn on Skin Wound Injury in Rats Accelerates the Wound Healing Process: Evidence from In Vitro and In Vivo Experimental Models" was published in 2022. Journal: Evid Based Complement Alternat Med.

[16] Al-Reza S. M., Rokonuzzaman M., Afroz M., Hussain M. I., Rashid M. A., Rahman A. (2016). Chemical composition and antioxidant activity of essential oil and organic extracts of Premna integrifolia Linn. *Brazilian Archives of Biology and Technology*.

[17] British Pharmacopoeia (BP) (1988). *Department of Health and Social Security Scottish Home and Health department*.

[18] OECD (2015). *Guideline for Testing of Chemicals: Draft Updated Test Guideline 434 on Acute Dermal Toxicity*.

[19] Nayak B. S., Anderson M., Pinto Pereira L. M. (2007). Evaluation of wound-healing potential of Catharanthus roseus leaf extract in rats. *Fitoterapia*.

[20] Kumar M. S., Kirubanandan S., Sripriya R., Sehgal P. K. (2008). Triphala promotes healing of infected full-thickness dermal wound. *Journal of Surgical Research*.

[21] Woessner J. F. (1961). The determination of hydroxyproline in tissue and protein samples containing small proportions of this imino acid. *Archives of Biochemistry and Biophysics*.

[22] Lowry O., Rosebrough N., Farr A. L., Randall R. (1951). Protein measurement with the Folin phenol reagent. *Journal of Biological Chemistry*.

[23] Singh M., Govindarajan R., Nath V., Rawat A. K. S., Mehrotra S. (2006). Antimicrobial, wound healing and antioxidant activity of Plagiochasma appendiculatum Lehm. et Lind. *Journal of Ethnopharmacology*.

[24] Gerlier D., Thomasset N. (1986). Use of MTT colorimetric assay to measure cell activation. *Journal of Immunological Methods*.

[25] Chen Y. (2012). Scratch wound healing assay. *Bio-protocol*.

[26] Clark R. A. F. (1985). Cutaneous tissue repair: basic biologic considerations. I. *Journal of the American Academy of Dermatology*.

[27] Kondo T., Ishida Y. (2010). Molecular pathology of wound healing. *Forensic Science International*.

[28] Bolla S. R., Mohammed Al-Subaie A., Yousuf Al-Jindan R. (2019). In vitro wound healing potency of methanolic leaf extract of Aristolochia saccata is possibly mediated by its stimulatory effect on collagen-1 expression. *Heliyon*.

[29] Sturtevant A. H. (1972). *Edible Plants of the World*.

[30] Lodhi S., Singhai A. K. (2013). Wound healing effect of flavonoid rich fraction and luteolin isolated from Martynia annua Linn. on streptozotocin induced diabetic rats. *Asian Pacific Journal of Tropical Medicine*.

[31] Li K., Diao Y., Zhang H. (2011). Tannin extracts from immature fruits of Terminalia chebula Fructus Retz. promote cutaneous wound healing in rats. *BMC Complementary and Alternative Medicine*.

[32] Gokani R. H., Lahiri S. K., Santani D. D., Shah M. B. (2011). Evaluation of anti-inflammatory and antioxidant activity of Premna integrifolia root. *Journal of Complementary and Integrative Medicine*.

The article "Topical Application of Premna integrifolia Linn on Skin Wound Injury in Rats Accelerates the Wound Healing Process: Evidence from In Vitro and In Vivo Experimental Models" was published in 2022. Journal: Evid Based Complement Alternat Med.

[33] Hassan S. W., Abubakar M. G., Umar R. A., Yakubu A. S., Maishanu H. M., Ayeni G. (2011). Pharmacological and toxicological properties of leaf extracts of kingelia africana (Bignoniaceae). *Journal of Pharmacology and Toxicology*.

[34] Ponrasu T., Suguna L. (2014). Efficacy of annona squamosa L in the synthesis of glycosaminoglycans and collagen during wound repair in streptozotocin induced diabetic rats. *BioMed Research International*.

[35] Puratchikody A., Devi C., Nagalakshmi G. (2006). Wound healing activity of cyperus rotundus linn. *Indian Journal of Pharmaceutical Sciences*.

[36] Yang J., Guo J., Yuan J. (2008). In vitro antioxidant properties of rutin. *Lebensmittel-Wissenschaft und -Technologie- Food Science and Technology*.

[37] Lodhi S., Jain A. P., Sharma V. K., Singhai A. K. (2013). Wound-healing effect of flavonoid-rich fraction fromTephrosia purpureaLinn. On streptozotocin-induced diabetic rats. *Journal of Herbs, Spices, & Medicinal Plants*.

[38] Udupa A. L., Kulkarni D. R., Udupa S. L. (1995). Effect of Tridax procumbens extracts on wound healing. *International Journal of Pharmacognosy*.

[39] Senthil Kumar M., Sripriya R., Vijaya Raghavan H., Sehgal P. K. (2006). Wound healing potential of Cassia fistula on infected albino rat model. *Journal of Surgical Research*.

[40] Rahman A., Sultana Shanta Z., Rashid M. A. (2016). In vitro antibacterial properties of essential oil and organic extracts of Premna integrifolia Linn. *Arabian Journal of Chemistry*.

[41] Mahnashi M. H., Alyami B. A., Alqahtani Y. S. (2021). Phytochemical profiling of bioactive compounds, anti-inflammatory and analgesic potentials of Habenaria digitata Lindl.: molecular docking based synergistic effect of the identified compounds. *Journal of Ethnopharmacology*.

[42] Sheriff Maqbul M., Alshabi A. M., Abdullatif Khan A. (2020). Comparative study of moringa oleifera with moringa peregrine seed oil using GC-MS and its antimicrobial activity against *Helicobacter pylori*. *Oriental Journal of Chemistry*.

[43] Abu-Dahab R. (2007). Antiproliferative activity of selected medicinal plants of Jordan against a breast adenocarcinoma cell line (MCF7). *Scientia Pharmaceutica*.

[44] Liang C.-C., Park A. Y., Guan J.-L. (2007). In vitro scratch assay: a convenient and inexpensive method for analysis of cell migration in vitro. *Nature Protocols*.

